# Application of Shewhart Control Chart in Controlling Adverse Events in Patients with Severe Acute Organophosphorus Pesticide Poisoning Undergoing Blood Purification

**DOI:** 10.1155/2022/9655423

**Published:** 2022-07-07

**Authors:** Zhen Zhang, Xufeng Mei, Qin Zhang

**Affiliations:** ^1^Blood Purification Centre, First People's Hospital of Linping District, Hangzhou, Zhejiang 311100, China; ^2^Department of Nephrology, First People's Hospital of Linping District, Hangzhou, Zhejiang 311100, China

## Abstract

**Objective:**

To explore the application effect of the Shewhart control chart in controlling adverse events in patients with severe acute organophosphorus pesticide poisoning (AOPP) undergoing blood purification.

**Methods:**

A retrospective analysis was performed on the clinical data of 102 patients with severe AOPP admitted to the hospital between January 2020 and December 2021, including 47 cases in the control group and 55 cases in the observation group. The control group was given routine emergency nursing, while the observation group was given emergency nursing under the guidance of the Shewhart control chart on the basis of the control group. The specialized operations, basic operations, specialized theory, and basic theory of nursing staffs were scored to compare the comprehensive nursing quality. The total incidence of adverse nursing events in both groups was statistically analyzed. The dosage of atropine, disappearance time of muscarinic symptoms, recovery time of CHE activity to 60%, and hospitalization time in both groups were recorded. The total incidence of complications in both groups was statistically analyzed. The satisfaction of family members was statistically analyzed by a satisfaction questionnaire.

**Results:**

The scores of specialized operations, basic operations, specialized theory, and basic theory of nursing staffs in the observation group were significantly higher than those in the control group (*P* < 0.05), total incidence of adverse nursing events was significantly lower than that in the control group (*P* < 0.05), dosage of atropine, disappearance time of muscarinic symptoms, recovery time of CHE activity to 60%, and hospitalization time were significantly lower than those in the control group (*P* < 0.05), total incidence of complications was significantly lower than that in the control group (*P* < 0.05), and scores of nursing attitude, communication process, psychological relief, and drug preparation were significantly higher than those in the control group (*P* < 0.05).

**Conclusion:**

The Shewhart control chart can effectively improve the clinical effect, comprehensive nursing quality, and satisfaction of patients with severe AOPP and effectively reduce complications and adverse events.

## 1. Introduction

Organophosphate pesticides (OPS) have been widely used in agricultural and forestry pest control worldwide since the 1930s due to their strong insecticidal effect and low cost [1]. However, in developing countries, especially in Asian countries, the lack of drug supervision and control often leads to acute organophosphorus pesticide poisoning (AOPP) [2]. AOPP is acute, with typical symptoms of salivation, sweating, pupil constriction, and muscle tremors. Critically ill patients also experience respiratory failure, disturbance of consciousness, shock, and death [3]. Timely and reasonable emergency nursing measures for severe AOPP patients can effectively shorten the rescue time and improve the success rate of rescue. In recent years, adverse events have occurred frequently in clinical nursing work. Adverse events mainly include the wrong drug administration, drug extravasation, falling from bed, falls, slippage of pipelines, and other potential safety hazard events other than their own diseases [4]. Therefore, how to establish a more effective and orderly emergency nursing program to ensure the quality of nursing and strengthen the management of adverse events, so as to improve the rescue effect and satisfaction of patients is a major challenge faced by the emergency department, and it is also a major challenge for emergency department nurses.

The Shewhart control chart was first proposed by Dr. Hasheart in 1924 and used in practical work. It refers to an image method that uses statistical techniques to control the measurement process, which can scientifically manage quality and accurately locate the problem and take timely solutions [5, 6]. With the rapid development of medical statistics and management, the Shewhart control chart is widely used in the field of infectious disease early warning in hospitals [7]. However, the Shewhart control chart is less used in patients with severe AOPP, and its application in nursing work is still in its infancy. Based on this, this study adopts the Shewhart control chart to manage the nursing quality of patients with severe AOPP and explore its application effect, in order to provide some ideas for improving the nursing effect of AOPP patients in the future.

## 2. Materials and Methods

### 2.1. General Data

A total of 102 severe AOPP patients admitted to our hospital from January 2020 to December 2021 were retrospectively selected as the research subjects. According to the admission time, 47 patients admitted to the hospital from January 2020 to December 2020 were divided into the control group. 55 patients admitted to the hospital from January 2021 to December 2021 were divided into the observation group. Inclusion criteria were (1) all patients were examined with severe AOPP, which met the relevant criteria in the “Clinical Expert Consensus on Diagnosis and Treatment of Acute Organophosphorus Pesticide Poisoning” [8]; (2) all patients were first organophosphorus poisoning; (3) patients' age ≥18 years old; (4) CHE activity ≤30%. Exclusion criteria were (1) the patient died during hospitalization; (2) the patient had nausea and tumor; (3) the patient had language or mental disorder; (4) the constitution was susceptible to drug allergy and coagulation dysfunction. There was no significant difference in general data such as gender, age, poisoning type, and the course of disease between the two groups (*P* > 0.05), and the results were comparable. As shown in Table 1.

### 2.2. Methods

The control group was given routine emergency nursing intervention; before admission, the nurses informed the patients or their family members about the way to induce vomiting by telephone and quickly induced vomiting. After the patients were admitted to the hospital, they immediately performed gastric lavage and drainage treatment. At the same time, venous blood was drawn from the patients to detect and analyze the types of toxic substances. The patients were treated with atropine, the patients with severe coma and respiratory failure were treated with pulmonary intubation ventilation to assist breathing, and the patients were treated with blood purification in the hemodialysis room. Afterwards, assist the doctor in the post-medication work, provide psychological counseling to the patient, give reasonable rehabilitation nursing care to control the diet, and instruct the patient and his family to cooperate with the doctor in the treatment, and strictly monitor the changes of patient's vital signs during the treatment.

On the basis of the control group, the observation group underwent emergency nursing intervention under the guidance of the Shewhart control chart. The specific implementation contents are as follows: (1) project monitoring: by reviewing the previous nursing records in our hospital and collecting statistics on adverse events in the nursing process of AOPP patients, it was found that the wrong drug administration, drug extravasation, falling from bed, falling, and slippage of the pipeline were all AOPP patients. Adverse events are common during nursing. Analyze the key factors that cause adverse events to determine whether the influence of this factor on the occurrence of adverse events is a key factor and whether there is a correlation with the usual daily management, and determine the negative impact of these adverse events after they occur. The main relevant items were monitored. It is necessary to focus on monitoring projects that may bring higher security risks or greater volatility. (2) The quality control is completed by the Shewhart control chart: the combination of the Shewhart control chart and the moving average method is used to determine the quality control standard. All data can be regarded as qualified within the control index, otherwise the data are considered to be unqualified. (3) Early-warning procedures: the early-warning system is set as the sequence, quality control chart, and typical cases. Sequence-based early-warning refers to early-warning of those factors that cause high incidence of adverse events. Ranking of incident factors were (1) poor work initiative and lack of sense of responsibility; (2) insufficient shift in shifts and weak inspection efforts; (3) insufficient operating skills and professional knowledge; Accurate; and (5) lack of communication skills. The top three factors should be prioritized for early warning, and then appropriate intervention measures should be formulated. For example, if falling from bed and falling, the ground needs to be kept dry, and patients and their families should be taught to prevent falls. If the drug is extravasated, the nursing staff needs to inform the patient in detail about the correct way of fixing the hand position and ask the family to supervise. When the pipeline slips, the nurses need to strengthen the inspection of the patient, communicate with the patient to prevent it from moving, and inform the patient of the risk of slippage when the patient is awake and try to let the patient cooperate. When the wrong medicine is given, the nursing staff needs to strictly follow the three checks and ten pairs to carry out the work, and the department needs to reasonably arrange the work according to the actual workload and working hours of each nursing staff to ensure sufficient manpower during the peak period. The quality control chart refers to predicting the risk range by setting specific procedures. If the data are within a reasonable range, the AOPP adverse event management work is considered to be effective; otherwise, corresponding adjustments should be made according to the actual situation. A typical case refers to the targeted early warning of the results, which is mainly based on the analysis of the harm caused by the adverse events of AOPP patients, combined with the patient's treatment process to review the auxiliary examination results to locate the fault links, as the basis for the prevention of such adverse events in the next stage, and provide a come up with a reasonable corresponding solution standard, so that the nursing staff can improve it according to the above standards.

### 2.3. Observation Indicators

1. Comprehensive nursing quality: the nursing staff is scored in the following four dimensions: specialized operation, basic operation, specialized theory, and basic theory. Each dimension has a full score of 100 points. Higher score indicates a better nursing quality.
2. The total incidence of adverse events in nursing: the number of adverse events such as wrong drug administration, drug extravasation, falling from bed, falling, and slippage of the pipeline were recorded during the intervention period.
3. Clinical effect: the dosage of atropine, the disappearance time of muscarinic symptoms, the time when cholinesterase (CHE) activity recovered to 60%, and the hospitalization time of the two patients were recorded.
4. The total incidence of complications: the total incidence of respiratory distress, organ dysfunction, stress bleeding, rebound, and other complications in the two groups was calculated.
5. Satisfaction: Satisfaction statistics of patients' family members were carried out using the self-made satisfaction questionnaire of the hospital. This table is divided into 4 dimensions including the nursing attitude, communication process, degree of psychological relief, and drug preparation, with 25 points for each item. The higher the score of each dimension, the higher the satisfaction.

### 2.4. Statistical Methods

SPSS 22.0 software was used for statistical analysis of the data. When the measurement data satisfies the normal distribution and the variance is homogeneous, it is expressed as ($\bar{x}\pm s$), the difference between the groups is compared by an independent *t* test, and the enumeration data are expressed by [*n* (%)], and the chi-square which is used for the comparison test <0.05 indicates statistical significance.

## 3. Results

### 3.1. The Comprehensive Quality of Nursing Scores in the Two Groups

The scores of specialized operation, basic operation, specialized theory, and basic theory in the observation group were significantly higher than those in the control group (*P* < 0.05), as shown in Table 2.

### 3.2. Comparison of the Incidence of Nursing Adverse Events between the Two Groups

During the intervention period, 2 (3.92%) cases of adverse events occurred in the observation group and 8 (15.69%) cases in the control group. The total incidence of adverse events in the observer was significantly lower than that in the control group (*P* < 0.05), as shown in Table 3.

### 3.3. Comparison of Clinical Effects between the Two Groups of Patients

The dosage of atropine, the disappearance time of muscarinic symptoms, the time for CHE activity to recover to 60%, and the time to discharge in the observation group were significantly lower than those in the control group (*P* < 0.05) as shown in Table 4.

### 3.4. Comparison of the Total Incidence of Complications between the Two Groups of Patients

There were 4 (7.84%) cases of complications in the observation group and 12 (23.53%) cases in the control group. The total incidence of complications in the observation group was significantly lower than that in the control group (*P* < 0.05) as shown in Table 5. All patients with complications received appropriate treatment and care.

### 3.5. Comparison of Nursing Satisfaction between the Two Groups

The observers' scores on the nursing attitude, communication process, psychological relief, and drug preparation were significantly higher than those in the control group (*P* < 0.05) as shown in Table 6.

## 4. Discussions

In clinical practice, AOPP is a common critical illness, which poses a serious threat to the life of patients due to its rapid onset and rapid changes in the condition [9]. Severe AOPP can lead to multiple organ failure, and clinical manifestations include respiratory failure, acute myocardial injury, cognitive impairment caused by nervous system damage, and decreased spatial learning ability. Blood purification therapy has been widely used in patients with severe AOPP and has achieved remarkable results [10]. Patients often experience symptoms of hypotension during hemodialysis treatment, and the incidence accounts for about 40% of all patients. Therefore, in the treatment of severe AOPP patients, it is of great clinical significance to improve the nursing quality of blood purification centers. The Shewhart control chart, also known as the quality management chart, analyzes and evaluates the stability of the implementation process according to the principles of mathematical statistics. Some quality management work has been applied, and its application value has been confirmed [11]. Using the Shewhart control chart to monitor nursing adverse events in real time and to strictly set the alert limit and control limit, one can effectively improve the level of nursing safety and quality management in clinical practice.

Some researchers [12] found that the Shewhart control chart can effectively warn of nursing risks, greatly reduce the incidence of adverse events in clinical nursing, and improve patients' satisfaction with nursing. Some researchers [13] believe that the early warning of adverse events reported through the quality control chart can greatly reduce the incidence of adverse events in the hospital and effectively improve the quality of care. The results of this study showed that after the application of the Shewhart control chart, the observation group was significantly better than the control group in terms of comprehensive nursing quality score, incidence of clinical adverse events, and patient satisfaction. The results of this study are partially similar to those reported in other articles [14]. The reason may be that when the Shewhart control chart is used for management and control, all adverse events are first set within the control range, and then the overall data is analyzed in detail. Targeted analysis is used to set the normal range of adverse events in the nursing process, so as to evaluate the probability of adverse events. Normal events are considered to be within the normal range, and those that exceed the normal range are considered to be adverse events. Then, the early warning of adverse events is carried out in sequence and typical cases. At the same time, it is necessary to carry out a comprehensive analysis based on the methods adopted in the clinic and provide effective data to accurately locate the link where the problem occurs. Finally, discussing the solution to the problem with experienced experts and formulating relevant countermeasures can effectively avoid the recurrence of similar events, thereby greatly reducing the incidence of adverse events for patients and reducing the risk of nursing care. The above strategies further ensure the safety of patients, maximize the interests of both doctors and patients, reduce the occurrence of conflicts, and ultimately achieve the purpose of improving the quality of care with the patient at the center.

The results of this study showed that the clinical effect of patients in the observation group was significantly better than that of the control group, and the complications were significantly lower than those in the control group. Evaluate, analyze, and designate improvement plans according to actual problems, and also use the statistical table method to monitor clinical nursing indicators in real time, which optimizes the quality of blood purification care to a certain extent. Therefore, the clinical effect of patients after blood purification treatment is improved, and concurrent symptoms were also reduced.

In conclusion, the application of the Shewhart control chart in patients with acute AOPP blood purification can effectively improve the clinical effect, comprehensive quality, and satisfaction of nursing and reduce adverse reactions and complications.

## Figures and Tables

**Table 1:** Comparison of general data of two groups of patients (*n*, $\bar{x}\pm s$).

Group	Number of cases	Gender (males/females)	Age (year)	Poisoning type				Disease duration
				Methamidophos	Dichlorvos	Trichlorfon	Dimethoate	
Control group	47	24/23	30.21 ± 4.22	17	11	8	11	2.58 ± 0.54
Observation group	55	30/25	31.05 ± 4.32	15	14	10	16	2.78 ± 0.64
*t*/*χ*^2^		0.123	0.989	1.012				1.689
*P*		0.725	0.325	0.798				0.094

**Table 2:** Comparison of the comprehensive nursing quality (*n*, $\bar{x}\pm s$, points).

Group	Number of cases	Specialist operation	Basic operation	Specialist theory	Basic theory
Control group	47	82.56 ± 3.54	84.21 ± 7.01	83.11 ± 5.14	84.08 ± 3.24
Observation group	55	87.56 ± 4.01	90.12 ± 9.54	88.65 ± 6.97	91.54 ± 5.68
*t*		6.622	3.512	4.501	7.962
*P*		<0.001	<0.001	<0.001	<0.001

**Table 3:** Occurrence of adverse events in the two groups of patients (*n*, %).

Group	Number of cases	Given wrong medicine	Drug extravasation	Falling out of bed	Falling down	Infusion line slippage	Total incidence
Control group	47	1 (2.13)	2 (4.26)	1 (2.13)	2 (4.26)	2 (4.29)	8 (17.02)
Observation group	55	0 (0.00)	0 (0.00)	1 (1.82)	1 (1.82)	0 (0.00)	2 (3.64)
*χ* ^*2*^							4.581
*P*							0.032

**Table 4:** Comparison of relevant indicators of the clinical effect (*n*, $\bar{x}\pm s$).

Group	Number of cases	Dosage of atropine (mg)	The time to disappearance of muscarinic symptoms (min)	Time to CHE activity recovers to 60% (h)	Hospitalizatio*n* time (d)
Control group	47	348.54 ± 77.65	20.11 ± 2.31	174.87 ± 30.21	14.02 ± 2.78
Observation group	55	284.56 ± 62.35	17.12 ± 2.01	154.68 ± 28.84	12.56 ± 2.24
*t*		4.614	6.991	3.448	2.937
*P*		<0.001	<0.001	0.001	0.004

**Table 5:** Complications in the two groups of patients (*n*, %).

Group	Number of cases	Respiratory distress	Organ dysfunction	Stress hemorrhage	Rebound phenomenon	Total incidence
Control group	47	3 (6.38)	2 (4.26)	2 (4.26)	3 (6.38)	10 (21.28)
Observation group	55	1 (1.82)	1 (1.82)	2 (3.64)	0 (0.00)	4 (7.27)
*χ* ^*2*^						4.197
*P*						0.040

**Table 6:** Comparison of two patients' satisfaction (*n*, %).

Group	Number of cases	Nursing attitude	Communication process	Degree of psychological relief	Drug preparation
Control group	47	17.01 ± 2.14	17.98 ± 2.04	15.11 ± 1.95	16.21 ± 2.01
Observation group	55	21.54 ± 3.33	20.64 ± 3.22	18.65 ± 2.66	19.39 ± 2.11
*t*		8.015	4.885	7.551	7.754
*P*		<0.001	<0.001	<0.001	<0.001

## Data Availability

The raw data supporting the conclusion of this article will be available from the corresponding author without undue reservation.
